# Implementation of Snow and Ice Sports Health and Sports Information Collection System Based on Internet of Things

**DOI:** 10.1155/2022/7411955

**Published:** 2022-01-07

**Authors:** Long Cheng

**Affiliations:** Zhengzhou University of Technology, Zhengzhou, Henan 450044, China

## Abstract

The promotion of ice and snow sports not only provides professional athletes for the Winter Olympics but also acts as appreciative mass bases for ice and snow sports. The appearance of ice and snow sports will bring a new consumption pattern and develop a new ice and snow industry. In this paper, an Internet of Things (IoT)-based sports information collection system which is specifically designed and developed for the healthcare domain specifically in the snow and ice sports is proposed. The physiological parameters such as body temperature, ECG, blood pressure, blood sugar, and blood oxygen saturation are captured through various monitoring devices. These physiological parameters are transmitted to the mobile device by the wireless module and mobile device that receives and displays these physiological parameters. A complete hardware design of the whole ice and snow sports health and sports information acquisition system, which is based on the Internet of Things, is given, and then, there is the overall design scheme of the system, such as adopted modular design for the system, attitude measurement unit, UWB positioning unit, data storage, and communication unit, respectively. The measurement results of the professional medical equipment are compared with those of acquisition equipment in real environment of ice and sports. These results have verified accuracy of data collected by acquisition equipment and meet the design requirements of the proposed system.

## 1. Introduction

With the enhancement of people's health awareness, national fitness has become a necessary means for healthy China. As a way of national fitness, ice and snow sports bring you a new experience in a new form of sports [1]. For ordinary athletes, real-time monitoring of their health and exercise status can help people adjust their exercise intensity or amount in time according to their daily exercise situation, so as to avoid physical discomfort caused by excessive or too little exercise and remind themselves to improve their exercise status in a timely manner and maintain a healthy body and a healthy life [2].

Maintaining a healthy body requires not only reasonable diet, but also scientific exercise habits [3]. A large number of studies have proved that regular aerobic exercise is beneficial to human health and can improve the exercise ability and physical quality of human body. In terms of health results and effectiveness of intervention programs, accurate quantification of physical exercise and physical health is very important [4–6]. Document [7] proposed the design and implementation of mobile medical monitoring client on Android platform. Document [8] designed and implemented a set of mobile Internet multiparameter health monitoring service systems to realize multiparameter measurement. Literature [9, 10] puts forward an open and reconfigurable wireless sensor network, which can transmit ECG, blood oxygen saturation SpO2, pulse wave, and other data amounts to remote service stations with different equipment configurations according to different diseases at different stages. Literature [11] uses piezoresistive triaxle acceleration sensor to measure the relationship between human motion acceleration and energy consumption. The acceleration of human body in daily activities such as sitting and walking can be measured, and then the relationship between acceleration value and energy consumption of human body movement can be obtained through experiments. Literature [12] proposes the fact that the acceleration sensor is fixed on the leg and the acceleration sensor can automatically detect the posture when the fibular nerve is stimulated and then analyze the walking posture of people. The system developed in [13, 14] can collect and analyze the movement posture of runners and give visual warning to incorrect movement forms. Literature [15] considers the complexity of athletes' sports process and establishes an accurate and flexible motion capture system, which can customize large sports venues covering multiple athletes and small movements of individual athletes, and is widely used in basketball, running, golf, high jump, and other sports, collecting athletes' sports information and providing objective data support for coaching courses.

In this paper, an Internet of Things (IoT) enabled sports information collection or capturing system, which is specifically designed and developed for the healthcare domain particularly in the snow and ice sports, is presented. For this purpose, various physiological parameters which are used during the experimental setup are body temperature, ECG, blood pressure, blood sugar, and blood oxygen saturation are captured through various monitoring devices. The major scientific contributions of this paper are provided as follows:

- A technology based automatic monitoring system for sports
- An Internet of Things enabled system which has the capacity of automatically monitoring the health status of various players in ice and snow sports
- A sophisticated mechanism, for both software and hardware related to health examination in the market at present, proposed to evaluate the effectiveness of the proposed mechanism in resolving the aforementioned issues
- Design and development of a health management system which includes the communication protocol for the wireless transmission of data from sensor, mobile devices, and cloud server devices.

The rest of the paper is arranged according to the following agenda items.

In the subsequent section, that is, Section 2, the proposed Internet of Things-based monitoring system is presented along with the overall framework.

## 2. Proposed Method: Internet of Things-Based System for ICE and Snow Sports

### 2.1. Overall System Framework

The physiological signal acquisition module and Bluetooth wireless communication module are integrated to complete data acquisition and transmission. The mobile program is developed based on Android platform, and the cloud server uses Apache and Nginx to build a high performance server. The overall framework design is shown in Figure 1.

Hardware acquisition equipment includes many modules such as blood pressure, blood oxygen, and ECG, which are responsible for the acquisition of user-related parameters. According to the data collection characteristics of the collection module, the transmission protocol of the module is designed, so that the wireless collection equipment can complete the mutual data transmission with the upper computer equipment [16]. At the same time, the upper computer completes the noise removal and display processing of the collected related data and displays the processed data visually in real time.

The cloud service platform receives the data sent by the mobile device and WIFI module via HTTP protocol and, at the same time, establishes a user-friendly WEB interactive page and designs related functions such as personal registration, login, and information consultation. The Redis and MySQL databases are used to store the data sent by the mobile platform. The combination of the two databases can persist and extract the physiological parameters of users and cope with the frequent insertion and extraction of data.

Finally, through the microservice framework with DUBBO as the core, the mutual call between internal and external systems is solved, which alleviates the pressure of high performance of the server to a certain extent and completes the related tasks of snow and ice sports health and sports information collection system.

### 2.2. Database Design

Real-time recording and saving of users' sports information not only are the needs of users themselves, but also help coaches to check the athletes' sports information and give some guidance according to their feedback information in time. With the increase of users, the amount of data in the system will also increase, which requires the effective management of users' movement information, so it is valuable to design a reasonable database to manage users' information [17, 18].

According to relevant rules, the logical relationship between database entities can be determined, which is the basis of database design. According to the three aspects of the system function, it can be concluded that the entities in the system are administrator entity, coach entity, and athlete entity. E-R diagram is used to describe the entity of athletes as shown in Figure 2.

The database includes five tables: general user information table, administrator information table, coach information table, feedback information table, and sports information table. In this paper, SQL server is chosen as the development environment for database design. First, tables and database diagrams are established, and then the database is read and written. Database operations use ADO.NET components, which, as a part of the. NET framework, provide classes for database operations. ADO.NET has two ways to read and write data: one is to use data providers; second is to use dataset.

The data acquired by dataset from the database is stored in the local memory, so it is necessary to keep the connection with the database all the time [19]. When an application needs data, it can directly read and modify the data from the dataset in memory and then write the modified data back to the database. In this paper, aiming at XP system, firstly IIS is installed in the local computer, then a new virtual host is created, and finally a website is added to the virtual host.

### 2.3. Hardware Design of the Human Motion Information Acquisition System

According to the requirements of the practical application of the system, the hardware structure of the system is designed. The hardware design of the system is mainly divided into the hardware design of attitude measurement unit, UWB indoor positioning unit, and data storage and communication unit [20]. Attitude measurement unit is the core measurement unit, and data storage and communication unit is the core communication unit. These two units are particularly important for human motion information acquisition system. UWB indoor positioning unit is an auxiliary function expansion unit. Combining this unit with attitude measurement unit can improve the positioning accuracy of the system and further improve the accuracy of motion information acquisition, which is of great significance in practical sports applications. The hardware structure diagram of the system is shown in Figure 3.

#### 2.3.1. Attitude Measurement Unit

Attitude measurement unit is the most important part of the system, which mainly includes MEMS sensors such as MEMS accelerometer, MEMS gyroscope and MEMS magnetometer, and microprocessor chip. In view of the possible miniaturization or high precision in practical application and the difference of installation and wearing position, two kinds of attitude measurement units are designed, namely, miniature attitude measurement unit and multifunctional attitude measurement unit.

The multifunctional attitude measurement unit has low requirements on volume, so MEMS sensors with higher accuracy can be selected. In order to achieve better expansion functions, microprocessor chips with stronger computing power, larger Flash storage space, and more peripheral interfaces can be selected. In this case, the MEMS sensor of the multifunctional attitude measurement unit selects three-axis accelerometer ADXL355, three single-axis gyroscopes ADXRS453, and three-axis magnetometer AK09970N, while the processor chip selects STM32F407VGT6. The hardware design of this scheme is shown in Figure 4.

The three MEMS sensors selected by the unit all support SPI communication, and the three-axis accelerometer ADXL355 and the single-axis gyroscope ADXRS453 have the same communication timing and phase. These two MEMS sensors can be directly connected with the SPI interface on the microprocessor chip. By using the chip selection signal, the time-sharing multiplexing function of the three MEMS sensors to SPI bus can be realized, thus realizing the high-speed collection function of the output of the three MEMS sensors, so that the microprocessor chip can process the data in real time.

#### 2.3.2. Positioning Unit

The UWB positioning unit is an auxiliary unit in the system, which can be selected when it is necessary to realize indoor and outdoor high-precision positioning functions. The unit mainly includes UWB chip, microprocessor chip, and communication antenna. The UWB chip is mainly responsible for sending and receiving data through the communication antenna, while the microprocessor chip is mainly responsible for calculating the distance and relative position between units by using UWB positioning algorithm, thus realizing indoor positioning function [21].

Using UWB technology, indoor and outdoor positioning functions can be realized. In order to achieve higher positioning accuracy, it is necessary to have certain preconditions; that is, there must be a certain number of UWB positioning base stations with known coordinate positions. Set in the three-dimensional spatial coordinate system *o* − *xyz*, the coordinates of the three positioning base stations are *B*_1_(*x*_1_, *y*_1_, *z*_1_), *B*_2_(*x*_2_, *y*_2_, *z*_2_), *B*_3_(*x*_3_, *y*_3_, *z*_3_), and the coordinates of the mobile tag are *T*(*x*, *y*, *z*); the locating base station *B*_1_ detects the included angle between the mobile tag *T* signal and the *z* axis that is *θ*_1_, and the locating base station *B*_2_ detects the included angle between the mobile tag *T* signal and the *x* axis that is *θ*_2_. The location base station *B*_3_ detects the included angle between the *T* signal of the mobile tag and the *y* axis that is *θ*_3_.

The geometric relationship between three positioning base stations and mobile tags can be obtained by using the above three-angle information. Equations established by geometric relations are shown in the following formula:

(1) $$\begin{array}{c} \left\{\begin{array}{c} \tan\;\theta_{1}=\frac{L}{z-z_{1}},\\ \tan\;\theta_{2}=\frac{x-x_{2}}{y-y_{2}},\\ \tan\;\theta_{3}=\frac{x-x_{3}}{y-y_{3}},\\ L=\sqrt{{\left(x-x_{1}\right)}^{2}+{\left(y-y_{1}\right)}^{2}}. \end{array}\right. \end{array}$$

Assuming that the real position coordinate of the mobile tag *T* is (*x*, *y*, *z*) and the estimated coordinate obtained by the positioning algorithm is $\left(\hat{x},\hat{y},\hat{z}\right)$, the mean square error (MSE) and root mean square error (RMSE) can be expressed as

(2) $$\begin{array}{c} \text{MSE}=E\left[{\left(\hat{x}-x\right)}^{2}+{\left(\hat{y}-y\right)}^{2}+{\left(\hat{z}-z\right)}^{2}\right],\\ \text{RMSE}=\sqrt{E\left[{\left(\hat{x}-x\right)}^{2}+{\left(\hat{y}-y\right)}^{2}+{\left(\hat{z}-z\right)}^{2}\right]}. \end{array}$$

Formula (2) can be used to estimate the position coordinates of mobile tags in three-dimensional space.

In the UWB positioning unit, MPU9250, a nine-axis motion sensor, is also selected as an auxiliary chip, which can realize the function of real-time judgment of the motion state of the unit. When the unit is set as a motion tag instead of a base station, if the nine-axis motion sensor MPU9250 detects the unit that is in a static state, the microprocessor chip will correspondingly send instructions to change the working state of the UWB chip in the unit, thereby reducing the working power consumption of the unit.

#### 2.3.3. Data Storage and Communication Unit

The data storage and communication unit is mainly responsible for storing and sending the attitude and motion information collected by each attitude measurement unit. The unit is mainly divided into an attitude data storage unit and a Bluetooth communication unit according to different practical application requirements. The attitude data storage unit can store the attitude and motion information collected by the attitude measurement unit into the memory card when the amount of data is too large or real-time calculation is unnecessary, and offline data processing can be performed at this time.

In the ice and snow sports health and sports information collection system based on Internet of Things, besides the attitude measurement unit which is responsible for collecting attitude and sports information, it also needs the data storage and communication unit to realize the functions of sending and storing the attitude and sports information collected by the attitude measurement unit. This unit can reduce the computational burden of microprocessor chip in the attitude measurement unit and avoid the impact on the real-time performance of information acquisition of the attitude measurement unit. The unit is mainly divided into two parts, namely, an offline data storage unit and a Bluetooth remote communication unit. The structural design of the data storage and communication unit is shown in Figure 5.

### 2.4. Software Design of the State Information Acquisition System

#### 2.4.1. Software Design of the Data Acquisition Node

Data acquisition nodes mainly include receiving data memory commands, collecting sensor data regularly and storing it in off-chip Flash, and uploading data. Considering the convenience of program development, the embedded software of data acquisition node does not introduce real-time operating system but adopts bare-metal program. Bare-metal programs are generally composed of a while loop in a main function and various interrupt service programs. The CPU executes the code in the while loop most of the time. When an interrupt event occurs, the CPU turns to execute the interrupt service program.

If the command to start collecting is received, the sensor data will be collected and stored in the off-chip Flash. After completing the acquisition and storage of one frame of data, it will be judged whether the command to end the acquisition sent by the data storage has been received, and if so, the acquisition will be stopped; otherwise, the acquisition will continue. After the acquisition is stopped, the data acquisition node will receive the upload command, read the sensor data from the off-chip Flash, and upload it to the data memory.

Inertial sensor unit provides two different ways to acquire sensor data: single register mode and burst register mode. Because this design only needs the data of acceleration, gyroscope, and magnetometer, and the data of all readable registers can be read once in burst mode, the single register mode is adopted. The read operation in single register mode requires two 16-bit SPI cycles. The address of the register to be read is input in the first cycle, and the value of the register to be read in the first cycle is output in the second cycle.  Figure 6 shows the read operation of three consecutive registers.

The host computer of the signal acquisition unit completes the functions of summarizing and uploading all signals. The host computer can upload the converted data in real time or regularly according to the preset functions. The preset functions are completed by pressing buttons. The flow chart of the host computer program is shown in Figure 7.

The initialization of the system after power-on mainly includes the initialization of the port and register of the MCU itself and the initialization of the Bluetooth module.

Because the master and slave of the signal acquisition unit are completed by 8-bit single chip microcomputer, and the time requirement of signal acquisition is high, no complex algorithm is involved in the program of the signal acquisition unit, and the signal filtering process is completed by the data processing link.

The data acquisition node starts the timer, and the timing time is 5 ms. If the response signal is not received within 5 ms, the previous data packet will be retransmitted. If the data receiving success command returning from the data memory is received, the new data packet is read from Flash and uploaded until all the collected data are uploaded. If the data is received by the data memory, but the return response signal is lost, the data will be received repeatedly, which will not affect the analysis result, because the data packets with the same data packet number will be ignored in the calculation process of gait parameters.

#### 2.4.2. Programming of the Data Processing Unit

The data processing unit mainly completes the following functions: after receiving acceleration data, the signal acquisition unit digitally filters it and uses reasonable algorithms to analyze and process the data to obtain relevant conclusions; Communication with the host computer, etc., and its software flow chart is shown in Figure 8.

In the system initialization, the ARM7 chip itself and related peripheral devices are initialized to ensure that each link is in normal working condition. After the initialization of the system, query and wait for the signal acquisition unit to upload the ready signal. If the system waiting time is exceeded, the system will try to communicate with the acquisition unit again. If the communication fails, the system will enter the standby state.

After the system completes initialization, the user can set relevant functions and parameters through the function buttons of the data processing unit, and the system will save the current settings. If the functions are not set, the system defaults to the last settings. The main significance of setting functions and parameters lies in the fact that acceleration sensors may be applied in different occasions, such as action normative judgment, movement speed measurement, and displacement measurement. The accuracy and algorithm will be different for different applications, so it is necessary to set functions and parameters.

In this system, the method of amplitude limiting filtering is adopted, that is, the two adjacent sampling values are subtracted, and the increment (expressed in absolute value) is calculated and then compared with the maximum allowable difference (determined by the actual situation of the collected object) Δ*Y* of the two samples. If it is less than or equal to Δ*Y*, the current sampling value is taken. If it is greater than Δ*Y*, the last sampling value is still taken as the current sampling value. That is,

(3) $$\begin{array}{c} Y=\left\{\begin{array}{c} Y\left(K\right),\left|Y\left(K\right)-Y\left(K-1\right)\right|\leq \Delta Y,\\ Y\left(K-1\right),\left|Y\left(K\right)-Y\left(K-1\right)\right|>\Delta Y. \end{array}\right. \end{array}$$

In different sports events, the acceleration changes of limb movements monitored by them may have great differences, and the acceleration and the rate of change of acceleration during movement at different test points of limbs are also different. The value of Δ*Y* also changes, so the value of Δ*Y* is obtained according to a large number of experiments and can be input through the keyboard when setting the system functions.

### 2.5. Noise Processing of Physiological Waveform Data

In the ice and snow sports health and sports information collection system based on the Internet of Things, for example, we need to obtain the final results of the measuring equipment, while the pulse wave signal and ECG signal may be interfered in the transmission process, resulting in incorrect measurement results. Therefore, in order to measure the accuracy and reliability of the results, it is necessary to do noise processing on the transmission waveform.

At the end of 20th century, Professor Norden E. Huang and others put forward the concept of Intrinsic Mode Function (IMF). EMD can be used to decompose signals to obtain a series of IMF. Every IMF must meet two requirements:

1. The number of zeros and poles in IMF components is equal or at most different by 1
2. The signal is symmetric about time axis

EMD is a processing method that decomposes the nonstationary pulse wave signal into several IMF component signals.

EMD decomposition steps are as follows:

(1) Find all local maxima and minima of signal *x*(*t*) and use cubic spline function to find the local mean of upper envelope *e*_max_ and lower envelope *e*_min_.
(2) All data centers contained in the two envelopes are marked *m*(*t*).
  (4) $$\begin{array}{c} m\left(t\right)=\frac{1}{2}\left(e_{\max}+e_{\min}\right). \end{array}$$
(3) Set *h*(*t*)=*x*(*t*) − *m*(*t*); calculate whether *h*(*t*) meets IMF conditions; if not, set it as new *x*(*t*), and continue step 2; otherwise repeat it *k* times.
  (5) $$\begin{array}{c} h_{1k}\left(t\right)=h_{k-1}\left(t\right)-m_{k}\left(t\right). \end{array}$$
In actual operation, the standard deviation *S* (*s* = 0.2 or 0.3) is taken as the standard to stop the cycle.
  (6) $$\begin{array}{c} S={\overset{T}{\underset{t=0}{\sum }}\left[\frac{h_{1\left(k-1\right)}\left(t\right)-h_{1k}\left(t\right)}{h_{1\left(k-1\right)}\left(t\right)}\right]}^{2}. \end{array}$$
(4) Through the above process, the IMF1 component *C*_1_=*h*_1*k*_(*t*) and the remaining items after separating the IMF1 component are obtained:
  (7) $$\begin{array}{c} r_{1}\left(t\right)=x\left(t\right)-C_{1}. \end{array}$$
(5) Continue to filter *r*_1_(*t*) according to the above steps and then get IMF2, IMF3... until *r*_*i*_(*t*) shows a monotonic trend or the value of *r*_*i*_(*t*) is very small; then stop the filter.

After the above five steps, the original signal can be reconstructed as follows:

(8) $$\begin{array}{c} x\left(t\right)=\overset{n}{\underset{i=1}{\sum }}C_{i}+r_{n}\left(t\right). \end{array}$$

EMD algorithm can deal with the adaptive denoising of nonstationary signals well and has better effect than Fourier transform and wavelet transform in nonstationary signal processing.

The processing mode of the upper computer of the sports health and sports information acquisition system is mainly the following process: the thread in charge of receiving waveform data in the upper computer receives the data and transmits it to the relevant waveform noise processing thread according to the waveform data category. When the noise thread is processed, the mobile client will display the processed data waveform on the interface, and the receiving thread in the cloud server will also display the waveform data on the WEB interface in real time and, at the same time, persist the processed noise waveform data in the database for subsequent query and diagnosis. The processing diagram is shown in Figure 9.

## 3. Result Analysis and Discussion

### 3.1. Bluetooth Connection Test

Use hardware to connect devices and check the time taken for successful connection after the simultaneous connection of multiple Bluetooth devices. Because the equipment used and the experimental process are basically similar to those in the previous section, you can see whether this connection is successful or not and the time elapsed from triggering the connection to the successful connection program in Android devices.

There are 100 groups of experiments in this experiment, including the total number of Bluetooth connections, Bluetooth connection time, total time of multiple Bluetooth connections, and average connection success time. The experimental data is shown in Figure 10.

It can be seen from Figure 10 that the number of connections can only be seven and the time for seven Bluetooth connections is gradually increasing. When connecting the eighth Bluetooth, the system will disconnect a Bluetooth that was successfully connected before and connect the eighth Bluetooth device at the same time, which takes a long time. Similarly, when the number of Bluetooth connections is seven, it takes 7.6 s in total and 1.13 s per connection on average. Time consuming is within the acceptable range, and multiple Bluetooth connections can be guaranteed at the same time.

### 3.2. Equipment Measurement Accuracy Experiment

On the one hand, it detects whether the results of multiple measurements by wireless health collection equipment are quite different; on the other hand, there is a big difference between the values of normal people and patients measured by health collection equipment. If these two aspects can be ensured within the error range, then this experiment can show that the measurement accuracy of wireless acquisition equipment is true and effective. Criterion uses variance to determine the degree of stability.

This test mainly depends on whether the measurement of acquisition equipment is stable. This experiment is a total of 100 times. The parameters tested include body temperature, blood sugar, blood pressure, heart rate, and blood oxygen. Blood sugar is measured on an empty stomach, while others are measured in a normal state.

Figures 11 and 12 show the measurement results of five kinds of measuring devices 100. It can be seen from the figures that the difference of multiple measurements is not very large.  Table 1 shows the variance of 100 measurement results of the same equipment. If the variance is smaller, the measured data is relatively stable. From the table, it can be seen that the variance of 100 measurement results of all measuring equipment is less than 0.5 and the one with higher volatility belongs to blood pressure, which may be due to body movement during the measurement. Therefore, this experiment can show that the wireless acquisition equipment runs stably and can provide good measurement services.

### 3.3. Accuracy Test of the Attitude Measurement Unit

Attitude measurement unit is the most critical part of the snow and ice sports health and sports information collection system based on Internet of Things, and the performance of attitude measurement unit directly affects the functions of the whole system. The MEMS accelerometer and MEMS gyroscope in the attitude measurement unit are independently calibrated by using a high-precision three-axis turntable, and the static and dynamic measurement accuracy of the calibrated attitude measurement unit are tested and verified.

In order to ensure the measurement accuracy of the system, MTi-G-710 inertial unit of Xsense Company is selected as a comparative reference to test the dynamic performance of the attitude measurement unit. The output data of MTi-G-710 can include accelerometer output, gyroscope output, and attitude angle output. In order to verify the dynamic attitude estimation accuracy of attitude measurement unit, the attitude angle is used as the comparison data, and the MTi-G-710 and attitude measurement unit output pitch angle, roll angle, and azimuth angle data under the same movement condition. The comparison test results are shown in Figures 13–15.

Through the static measurement accuracy test of the attitude measurement unit in the ice and snow sports health and sports information acquisition system based on the Internet of Things and the dynamic accuracy test compared with MTi-G-710 inertial group, the characteristics of small size and high accuracy of the attitude measurement unit are fully reflected, and the test results are consistent with the MATLAB simulation results, which fully verifies the effectiveness of the omnidirectional attitude estimation algorithm.

### 3.4. Positioning Accuracy Test

The location algorithm based on UWB technology is given above, and a UWB location unit based on DW1000 chip is designed. This part will test the location accuracy of UWB location unit. In the test, Chan's algorithm based on TDOA is used to calculate the coordinate position of mobile tag. In the actual test process, because the real-time motion trajectory of UWB positioning unit is difficult to measure, several discrete points with known coordinates of relative positioning base stations are selected as test points to test the positioning accuracy of UWB positioning unit.

From Figure 16, we can analyze the positioning errors of UWB in five positioning base stations more intuitively. From the figure, we can see that the positioning errors of UWB in *z* axis direction are obviously suppressed, while the errors in other two coordinate axes and distance errors are suppressed, and the errors in *x* axis direction and *y* axis direction can be controlled within 0.2 m.

Based on the above results, the accuracy of using Chan's algorithm based on TDOA to realize UWB positioning function is verified. By increasing the number of positioning base stations, the positioning accuracy of the system is effectively improved, and the information collection accuracy of the ice and snow sports health and sports information collection system based on Internet of Things is fully guaranteed.

## 4. Conclusion

Under the background of China's health strategy, snow and ice sports are proposed because health is the product of social development at a certain stage. With the improvement of people's living standards, people will pay more and more attention to health. This paper mainly completes the research of snow and ice sports health and sports information collection system based on the Internet of Things, including the related integration of wireless communication module and collection equipment, the design of wireless transmission protocol and related analysis, and program design of mobile platform and high performance cloud server. In order to solve the problem that MEMS sensors are easily affected by ambient temperature, temperature compensation is carried out for MEMS sensors. According to the requirement of UWB positioning, the common UWB positioning algorithms are analyzed, and their positioning accuracy is verified by simulation; thus the main algorithms in the snow and ice sports health and sports information collection system based on Internet of Things are given. The motion information collected by the system can reflect the characteristics of each action, which is convenient for subsequent identification and analysis. Through the test, the system has a good ability of collecting human motion information.

Although the ice and snow sports health and sports information collection system based on Internet of Things is running normally at present, there are still some shortcomings in the design and processing process, which need to be improved and solved later. There are some differences in the accuracy of physiological signal processing. Because the amount of data processed is a small sample, a large amount of hospital data may be needed to improve the accuracy of the algorithm.

## Figures and Tables

**Figure 1:** Overall framework design of sports health and sports information collection system.

**Figure 2:** E-R diagram of athletes.

**Figure 3:** Hardware structure diagram of ice and snow sports health information collection system based on Internet of Things.

**Figure 4:** Hardware design drawing of multifunctional attitude measurement unit.

**Figure 5:** Structural design drawing of the data storage and communication unit.

**Figure 6:** Example of SPI read operation of the inertial sensor.

**Figure 7:** Flow chart of signal acquisition unit host software.

**Figure 8:** Data processing unit software flow chart.

**Figure 9:** Schematic diagram of noise processing for sports health and sports information collection system.

**Figure 10:** Time-consuming statistics of multiple Bluetooth connections.

**Figure 11:** Blood pressure and blood oxygen measured 100 times.

**Figure 12:** Blood glucose, ear temperature, and ECG measured 100 times.

**Figure 13:** Comparison test results of pitch angle between attitude measurement unit and existing MTI inertial unit.

**Figure 14:** Comparison test results of roll angle between attitude measurement unit and existing MTI inertial unit.

**Figure 15:** Azimuth comparison test results between attitude measurement unit and existing MTI inertial unit.

**Figure 16:** Average error of UWB positioning of five positioning base stations.

**Table 1:** Multiple measurement variances of the same equipment.

Type	Hypertension	Hypotension	Blood sugar	Ear temperature	Blood oxygen	Heart rate
Variance	0.201	0.14	0.002	0.054	0	0.326

## Data Availability

The data used to support the findings of this study are included within the article.
